RETRACTED

# Corrective Efficacy of Calcaneal Lengthening Osteotomy for Planovalgus Deformity in Cerebral Palsy Patients

**DOI:** 10.7759/cureus.57092

**Published:** 2024-03-27

**Authors:** Vinod Dubey, Sohilkhan R Pathan, Dhruv Sharma

**Affiliations:** 1 Orthopaedic Surgery, Shree Krishna Hospital and Medical Research Centre, Pramukhswami Medical College, Bhaikaka University, Anand, IND; 2 Clinical Research Services (CRS), Bhanubhai and Madhuben Patel Cardiac Centre, Shree Krishna Hospital and Medical Research Centre, Anand, IND

**Keywords:** surgical correction, pediatric orthopedics, calcaneal lengthening osteotomy (clo), planovalgus deformity, cerebral palsy

## Abstract

Introduction

Planovalgus deformity is common in children with spastic cerebral palsy (CP), particularly spastic diplegia and spastic quadriplegia. It results from muscle imbalance over the immature foot skeleton, leading to hindfoot valgus, forefoot abduction, and joint subluxation. Surgical interventions, like calcaneal lengthening osteotomy (CLO), are frequently employed to correct this deformity, but objective guidelines for its use in CP patients are lacking.

Material and methods

This retrospective cohort study examined the efficacy of CLO in correcting plano valgus deformity in pediatric CP patients at the Pediatric Orthopedic Unit of Christian Medical College (CMC) in Vellore, India. Data from patient records and radiographs were collected, including demographics, pre- and postoperative angles, and surgical details. Statistical analysis was performed to assess changes in angles and associations with various factors.

Results

After the surgery, there was a notable enhancement in the calcaneal pitch, lateral talo-first metatarsal angle, and naviculocuboid overlap, as shown by the CLO results. However, tibiocalcaneal angles did not show significant changes. Associations were observed between age, Gross Motor Function Classification System (GMFCS) level, additional surgeries, and postoperative angle corrections.

Conclusion

CLO shows promise in correcting plano valgus deformity, with age, GMFCS level, and comorbidities influencing outcomes. Long-term follow-up is crucial to monitor correction durability. Specific radiographic angles provide insights into CLO's biomechanical effects, but study limitations warrant caution in interpretation. CLO effectively corrects plano valgus deformity in pediatric CP patients, with age, GMFCS level, and comorbidities influencing outcomes. Long-term follow-up and further research are needed to optimize management strategies and enhance understanding of surgical outcomes.

## Introduction

Planovalgus deformity is a very common deformity in children with spastic cerebral palsy (CP) especially spastic diplegia and spastic quadriplegia [1]. The deformity occurs most commonly due to muscle imbalance occurring over the skeletally immature foot [2]. It frequently leads to hindfoot valgus deformity and forefoot abduction, subluxation, and dislocation of the talonavicular and calcaneocuboid joint. Children's weight bears on the talus and navicular, which causes pain and callosity formation [3-4]. The talus subluxates toward the medial and plantar sides. Dorsiflexion and external rotation of calcaneus in relation to the talus and calcaneus in plantar flexion compared to the tibia. Further dysfunction of the lever arm is caused as the forefoot is supinated and externally rotated leading to lateral column shortening [5]. Many surgical procedures, like medial displacement osteotomy of the calcaneus, extra-articular arthrodesis, lateral column lengthening, and triple arthrodesis, have been described in the literature. Calcaneal lengthening osteotomy (CLO) has been used most commonly to correct the planovalgus deformity in CP children with moderate to severe types.

RETRACTED

Pes planus refers to the condition marked by the collapse of the medial longitudinal arch of the foot. When combined with heel valgus, it is termed pes planovalgus. This deformity is typified by several features: plantar flexion of the talus, outward rotation of the calcaneus relative to the talus resulting in the prominence of the talar head, pronounced eversion of the subtalar joint, displacement of the navicular bone in relation to the talar head, and supination of the forefoot with respect to the hindfoot [6-9]. Planovalgus foot deformity is commonly seen in diplegic and quadriplegic patients with CP. During a normal gait cycle, the length of the foot from the heel to the metatarsal head acts as a lever arm for the tendino-achilles. In CP patients with planovalgus deformity, the effective lever arm function of the foot is lost due to midfoot break, and the new shorter lever arm available during the push-off is from the heel to the midfoot. As a result, the muscles have to generate more amount of force to balance the ground reaction force. In addition, the defective lever arm prevents an adequate transfer of forces from the ground reaction force (GRF), which falls behind the knee, leading to knee flexion in the mid-stance phase, and the normal plantarflexion-knee hyperextension coupling is lost. This produces abnormal gait kinematics, which is manifested as increased knee flexion and internal rotation at the hip [10-11].

Conservative treatment can be tried in the form of bracing to anatomically realign the foot skeleton so that the progression of deformity can be stopped. Ground-reaction ankle foot orthosis (AFO) is a useful technique to restore the normal ankle plantarflexion-knee hyperextension coupling. Effective bracing with appropriate orthosis can improve foot lever arm function and restore the normal GRF moment anterior to the knee during walking. Surgical treatment is indicated for patients who no longer tolerate orthotics or when lever arm dysfunction interferes with function. Surgical procedures described include subtalar extraarticular arthrodesis, triple arthrodesis, and arthroereisis of the sinus tarsi [12-14]. CLO, initially introduced by Evans in 1975, underwent modifications by Mosca in 1995 [15-17].

RETRACTED

However, there is no specific objective guideline to perform CLO in planovalgus deformity in CP patients. Indications of any additional procedures, like medial talonavicular joint capsular tightening, arthrodesis of the medial column joints, lateral column joints, and triple arthrodesis, are not clearly defined in the literature.

## Materials and methods

Study design

The study utilized a retrospective cohort design to assess the effectiveness of CLO in correcting planovalgus deformity in pediatric patients diagnosed with CP. This design allows for the examination of outcomes over time by comparing a group of patients who received the intervention (CLO) with a control group or their own pre-intervention status.

Inclusion and exclusion criteria

Patients under 18 years of age diagnosed with CP, presenting with unilateral or bilateral plano valgus foot deformity, and who underwent CLO with or without additional procedures were included. In addition, patients needed to have a minimum follow-up period of one year post-operation and the availability of both preoperative and postoperative weight-bearing foot anteroposterior (AP) and lateral X-rays. Exclusion criteria comprised patients above 18 years of age, absence of CP diagnosis, presentation with foot deformities other than planovalgus, undergoing a different surgical intervention or no intervention, a follow-up period of less than one year post-operation, and unavailability of preoperative and postoperative X-rays.

Study population

A total of 18 patients were identified from records and radiographs obtained between June 2012 and June 2017 at the Pediatric Orthopedic Unit of Christian Medical College (CMC) in Vellore, India.

Data collection

Data were collected through a comprehensive review of patient records and radiographs. Relevant information included patient demographics, medical history, preoperative foot deformity characteristics, surgical details (including CLO procedure and any additional interventions), and postoperative outcomes. Preoperative and postoperative weight-bearing foot AP and lateral X-rays were used for assessing deformity correction and other relevant measures.

RETRACTED

Statistical analysis

Descriptive statistics summarized patient demographics, surgical procedures, and outcomes. Inferential statistics (paired t-test) determined preoperative vs. postoperative differences. Correlation analysis identified associations between variables. Regression analysis explored relationships between variables. 

Ethical details

The study was conducted in accordance with ethical guidelines and regulations. Ethical approval was obtained from the Institutional Review Board or Ethics Committee of CMC in Vellore. Patient confidentiality and privacy were maintained throughout the study, with data anonymized during analysis and reporting.

## Results

A total of 18 patients and 31 feet were included in the analysis. Of these patients, 11 were male, constituting over 60% of the study cohort, while the remaining seven were female. The average age of the children at the time of surgery was 13.3 years, with a standard deviation of 5.5 years, and the average follow-up period was 18.8 months, with a standard deviation of 6.7 months. Six patients were classified as Gross Motor Function Classification System (GMFCS) level 2, indicating mild to moderate functional impairment, while the remaining 12 patients belonged to GMFCS level 3, representing moderate to severe impairment. Approximately two-thirds of the patients fell within GMFCS level 3. Regarding surgical procedures, three patients underwent surgery on the medial side, while the remaining 15 patients underwent only CLO. Thus, 16.7% of the patients underwent additional surgery on the medial side, while the majority (83.7%) solely underwent CLO (Table 1).

**Table 1:** Distribution of patient characteristics ** Others include b/l medial cuneiform plantar closing wedge, left foot medial reefing, and right navicular medial closing wedge osteotomy. # Others include maternal DM, jaundice, and myelomeningocele. GMFCS: Gross Motor Function Classification System

Variables	n	%
Gender		
Male	11	61.1
Female	7	38.90
GMFCS level		
2	6	33.3
3	12	66.7
Medial side surgery		
Nil	15	83.3
Others **	3	16.7
Type of cerebral palsy		
Spastic diplegia	15	83.3
Spastic hemiparesis	1	5.6
Spastic quadriplegia	2	11.1
Other medical condition		
Nil	11	61.1
Seizure disorder	5	27.8
Others ^#^	2	11.1
	Mean ± SD	
Age	13.3 ± 5.5	
Follow-up surgery (in months)	18.8 ± 6.7	

In terms of CP subtype, the majority of patients were diagnosed with spastic diplegia (n = 15), while two patients had spastic quadriplegia and one patient had spastic hemiparesis. Among the 18 children included in the study, 12 did not have any comorbidities, while five had a history of seizures and one had a history of jaundice during the neonatal period. The calcaneal pitch demonstrated a statistically significant increase in both the right and left feet following the operation (p = 0.036 and p < 0.001, respectively). Specifically, the median preoperative and postoperative angles on the right side were 2.94 ± 10.38 and 9.40 ± 5.78 degrees, respectively, while on the left side, they were 3.06 ± 7.21 and 9.59 ± 3.57 degrees, respectively. The change in angle between preoperative and postoperative measurements was found to be statistically significant. Out of the 31 feet analyzed, 11 feet (35.48%) exhibited correction within the normal range for calcaneal angles postoperatively. This indicates a notable improvement in foot alignment following the surgical intervention (Table 2).

RETRACTED

**Table 2:** Descriptive statistics (paired t-test) and change in pre- and postoperative values for feet’s measurements.

Parameters	Preoperative	Postoperative	Mean difference	95% CI	p-value
	Mean ± SD	Mean ± SD			
Calcaneal pitch					
Right	2.94 ± 10.38	9.40 ± 5.98	-6.46	-12.45, -0.47	0.036
Left	3.06 ± 7.21	9.59 ± 3.57	-6.53	-9.46, -3.60	<0.001
Tibiocalcaneal angle					
Right	77.55 ± 13.93	72.78 ± 14.84	4.78	-1.23, 10.78	0.111
Left	73.94 ± 14.44	67.59 ± 19.81	6.36	-1.89, 14.60	0.121
Talo 1^st^ metatarsal angle					
Right	26.54 ± 18.71	19.01 ± 11.01	7.53	1.17, 13.88	0.023
Left	29.33 ± 15.25	21.61 ± 12.92	7.73	0.95, 14.50	0.028
Lateral talocalcaneal angle					
Right	38.35 ± 10.22	36.73 ± 9.81	1.63	-3.17, 6.42	0.481
Left	38.24 ± 10.98	40.65 ± 9.74	-2.41	-6.85, 2.03	0.265
Naviculocuboid overlap					
Right	0.83 ± 0.30	0.66 ± 0.39	0.17	0.05, 0.29	0.010
Left	0.83 ± 0.27	1.18 ± 1.78	-0.34	-1.29, 0.61	0.452
Metatarsal stacking angle					
Right	5.46 ± 5.64	8.59 ± 7.42	-3.13	-7.32, 1.07	0.133
Left	7.28 ± 8.13	7.58 ± 6.83	-0.30	-2.80, 2.20	0.802
Medial lateral column ratio					
Right	0.99 ± 0.09	0.98 ± 0.08	0.01	-0.04, 0.06	0.605
Left	1.02 ± 0.09	1.01 ± 0.07	0.01	-0.02, 0.05	0.467
Talonavicular coverage angle					
Right	30.60 ± 16.39	14.49 ± 11.19	17.17	6.03, 28.32	0.005
Left	34.89 ± 10.14	11.21 ± 11.64	24.47	15.49, 33.44	<0.001
1^st^ metatarsal talar angle					
Right	25.36 ± 14.74	16.08 ± 10.82	10.57	-0.56, 21.7	0.061
Left	25.29 ± 13.82	13.85 ± 8.36	12.84	2.39, 23.3	0.020

The mean preoperative and postoperative tibiocalcaneal angles on the right side were 77.55 and 72.78 degrees, respectively, while on the left side, they were 73.94 and 67.59 degrees, respectively. The mean differences between the preoperative and postoperative angles were 4.78 degrees on the right side and 6.36 degrees on the left side, although these differences were not found to be statistically significant. Despite a decrease in angle from preoperative values after surgery, the observed differences did not reach statistical significance. Among the 31 feet analyzed, 14 feet (45.16%) exhibited tibiocalcaneal angles within the normal range postoperatively (Figure 1).

RETRACTED

**Figure 1:** Preoperative calcaneal pitch (angle before surgery) and postoperative calcaneal pitch (angle after surgery).

Regarding the lateral talo-first metatarsal angles, the mean preoperative and postoperative values on the right side were 26.54 and 19.01 degrees, respectively, while on the left side, they were 29.33 and 21.61 degrees, respectively. The differences were found to be statistically significant. Specifically, nine feet (29%) achieved correction to the normal range postoperatively, indicating an improvement in foot alignment following the surgical intervention. 

The mean preoperative and postoperative lateral talocalcaneal angles on the right side were 38.35 and 36.73 degrees, respectively, while on the left side, they were 38.24 and 40.65 degrees, respectively. The observed differences were not statistically significant. However, postoperatively, 21 feet (67.74%) achieved correction to the normal range, indicating an improvement in foot alignment (Figure 2).

**Figure 2:** Lateral talo-first metatarsal angle preoperative (before surgery) and postoperative (after surgery).

Regarding the naviculocuboid overlap, the mean preoperative and postoperative values on the right side were 0.83 and 0.66, respectively, while on the left side, they were 0.83 and 1.18, respectively. The differences were found to be statistically significant on the left side but not on the right side. Postoperatively, 20 feet (64.51%) were corrected to the normal range, demonstrating a notable improvement in foot alignment following the surgical procedure (Figure 3).

**Figure 3:** Naviculocuboid overlap preoperative and postoperative.

The mean preoperative and postoperative metatarsal stacking angles on the right side were 5.46 and 8.59 degrees, respectively, while on the left side, they were 7.28 and 7.58 degrees, respectively. The observed differences were not statistically significant. However, postoperatively, 25 feet (80.64%) achieved correction to the normal range, indicating an improvement in foot alignment.

Similarly, the mean preoperative and postoperative medial-lateral column ratios on the right side were 0.99 and 0.98, respectively, while on the left side, they were 1.02 and 1.01, respectively. The observed differences were not statistically significant. Nevertheless, postoperatively, 29 feet (93.54%) were corrected to the normal range, suggesting an improvement in foot alignment.

RETRACTED

It is noteworthy that the lateral column lengthening between preoperative and postoperative measurements was found to be statistically significant on both sides, indicating a notable alteration in foot structure following the surgical intervention (Figure 4).

**Figure 4:** Medial lateral column ratio: preoperative and postoperative.

The mean preoperative and postoperative talo-navicular coverage angles on the right side were 30.60 and 14.49 degrees, respectively, while on the left side, they were 34.89 and 11.21 degrees, respectively. The observed differences were statistically significant on both sides. Following the operation, 20 feet (66.66%) achieved correction to the normal range, indicating an improvement in foot alignment (Figure 5).

**Figure 5:** Talo-navicular coverage angle preoperative and postoperative.

Similarly, the mean preoperative and postoperative AP talo-first metatarsal angles on the right side were 25.36 and 16.08 degrees, respectively, while on the left side, they were 25.29 and 13.85 degrees, respectively. The differences were found to be statistically significant on the left side. Postoperatively, 13 feet (43.33%) were corrected to the normal range, signifying an improvement in foot alignment (Figure 6).

**Figure 6:** Anteroposterior talo-first metatarsal angle preoperative and postoperative.

The correlation analysis revealed several noteworthy associations regarding the change in angles between preoperative and postoperative measurements. Older patients tended to experience a greater change in calcaneal pitch, possibly indicating more pronounced correction or worsening of deformity with age, although this association was not statistically significant. Conversely, an increase in follow-up duration was associated with a decrease in the difference in calcaneal pitch, suggesting potential insufficient correction over time. Moreover, patients with higher GMFCS levels had a greater change in calcaneal pitch, indicating more severe deformity requiring more correction. Interestingly, patients who underwent additional medial side surgeries had a decreased change in calcaneal pitch, possibly indicating inadequate correction. Furthermore, patients with more comorbidities, such as seizures, tended to have a greater difference in calcaneal pitch, suggesting more severe deformities or incomplete correction due to medical conditions.

The analysis of the tibiocalcaneal angle revealed several significant associations: As age increases, the difference in the tibiocalcaneal angle tends to decrease, suggesting incomplete correction or potential diminishment of the deformity over time, possibly influenced by concurrent knee-level deformities. In addition, the difference in the angle increases with each month of follow-up post-surgery, indicating a statistically significant trend potentially biased by knee joint correction. Higher GMFCS levels correspond to less correction, likely due to knee flexion contractures. Patients undergoing additional medial side surgery exhibit the most significant change in the angle, suggesting a significant influence of knee joint deformity correction. Medical conditions like seizures are associated with difficulty correcting the deformity, possibly due to the complexity of managing multiple medical issues concurrently.

RETRACTED

The analysis of the lateral talo-first metatarsal angle revealed several significant associations: Increasing age was associated with a decrease in the difference in angle, suggesting greater correction requirements in older children, possibly indicative of more severe deformities or increased difficulty in achieving normal alignment. Follow-up duration showed a positive association with the difference in angle, indicating sustained correction over time, reflecting the lasting effectiveness of corrective procedures. Higher GMFCS levels, particularly level 3, were linked to more severe deformities, suggesting challenges in achieving full correction. Children who underwent medial side surgery exhibited greater correction, highlighting the efficacy of additional surgical interventions. Conversely, comorbid conditions, such as seizure disorders, were associated with decreased correction, indicating challenges in achieving adequate alignment possibly due to the complexity of managing multiple medical issues or lesser deformities associated with comorbid conditions.

The analysis of the lateral talocalcaneal angle revealed several key findings: First, the difference in angle decreased with increasing age, indicating a greater need for correction in older children, potentially due to the progression or severity of the deformity. Second, longer follow-up durations were associated with increased correction or indication of more severe, uncorrectable deformities over time. Higher GMFCS levels correlated with greater correction requirements, suggesting challenges in fully correcting deformities in children with more severe functional impairments. The addition of medial side surgery showed a negative trend in the angle difference, suggesting that such surgeries may not fully correct deformities to the normal level. Moreover, comorbid conditions, including seizures, were associated with increased correction, implying more severe deformities or additional correction needed due to medical factors. Despite these associations, they were not statistically significant, likely influenced by other surgeries involved in single-event multilevel surgery (SEMLS) or deformities at the knee or hip regions.

RETRACTED

The analysis of naviculocuboid overlaps unveiled several significant associations: First, both age and follow-up duration correlated with an increase in deformity or the need for greater correction, suggesting that as children age and the follow-up period extends, deformities may progress, necessitating increased correction. Second, severe GMFCS levels were associated with more severe pronated feet and an inability to fully correct the deformity, indicating challenges in correcting complex deformities or achieving complete correction. Furthermore, additional medial side surgery, typically performed in cases of severe deformity, resulted in greater correction compared to cases without such surgery, suggesting its efficacy in addressing severe deformities. Conversely, the presence of other medical comorbid conditions had a negative impact on correction, complicating the correction process or making it more challenging to achieve satisfactory results. While these associations were observed, their significance was not specified, underscoring the multifactorial nature of naviculocuboid overlaps and the diverse factors influencing correction outcomes.

The analysis of the metatarsal stacking angle revealed significant associations: Age, follow-up duration since surgery, and GMFCS level showed positive correlations with an increase in the angle difference, indicating a greater need for correction in forefoot supination as children age, as follow-up duration increases, and as GMFCS level becomes more severe. In addition, medial-side surgery and other medical disorders were associated with increased forefoot supination, suggesting their contribution to persistent deformities beyond the normal range. Specifically, children with seizure disorders and those undergoing medial-side surgery exhibited more pronounced supination. Overall, while follow-up duration since surgery showed statistically significant results, emphasizing its impact on forefoot supination correction, these associations underscore the importance of considering age, follow-up duration, GMFCS level, and additional surgeries or medical conditions when addressing forefoot supination deformities.

The analysis of the medial-lateral column ratio revealed significant associations: Age, follow-up duration since surgery, GMFCS level, and other medical conditions were inversely correlated with the ratio, indicating an increase in the lateral column relative to the medial column with advancing age, longer follow-up duration, higher GMFCS levels, and the presence of medical conditions. Conversely, in cases with medial side surgery, the ratio increased, suggesting effective correction of medial column shortening. These findings emphasize the impact of age, follow-up duration, functional impairment level, and additional surgeries on the medial-lateral column ratio, underscoring their importance in deformity assessment and management.

RETRACTED

The analysis of the talonavicular coverage angle revealed significant associations: Age and GMFCS level exhibited a positive correlation with postoperative correction, indicating greater deformity severity in older children and those with higher GMFCS levels. In addition, children with seizure disorders required more correction, potentially due to the influence of seizures on muscle tone and motor function. Follow-up duration showed a negative association, suggesting a potential loss of correction over time. Moreover, cases with medial-side surgery exhibited decreased correction, emphasizing the importance of considering these factors in deformity management and postoperative outcomes.

The analysis of the AP first metatarsal talar angle revealed several significant associations. Age exhibited a positive correlation with the angle difference, suggesting increased correction needs in older children, possibly indicating more severe or progressive deformities. Conversely, follow-up duration, GMFCS level, medial-side surgery, and seizure disorders showed a negative correlation with the angle difference, indicating incomplete correction or severe, uncorrectable deformities in cases with longer follow-up duration, higher GMFCS levels, medial-side surgery, or seizure disorders. These findings underscore the complexity of factors influencing the AP first metatarsal talar angle and highlight the importance of personalized assessment and management strategies tailored to individual patient characteristics and deformity severity (Tables 3, 4, 5).

**Table 3:** Correlation between various angles and factors. In this representation, the upward arrow (↑) signifies a positive correlation, while the downward arrow (↓) denotes a negative correlation.

Surgical outcome	Calcaneal pitch	Tibiocalcaneal angle	Talo first metatarsal angle	Lateral talocalcaneal	Naviculo-uboid overlap	Metatarsal staking angle	Medial-lateral column ratio	Talonavicular coverage angle	Anteroposterior talo-first metatarsal angle
Age	↑	↓	↓	↓	↑	↑	↓	↑	↑
Postoperative monitoring	↓	↑	↑	↑	↑	↑	↓	↓	↓
GMFCS level	↑	↓	↑	↑	↓	↑	↓	↑	↓
Medial-side surgery	↓	↑	↑	↓	↑	↓	↑	↓	↓
Comorbidity evaluation	↑	↓	↓	↑	↓	↓	↓	↑ (Seizure disorders)	↓

**Table 4:** Random intercept model for the difference of parameters from the preoperative period to postoperative period GMFCS: Gross Motor Function Classification System

Variables	Coefficient	95% CI	p-value
Calcaneal pitch			
Age	0.68	-0.11, 1.48	0.094
Follow-up surgery	-0.27	-0.77, 0.24	0.301
GMFCS			
2 (ref)	0		
3	0.31	-8.33, 7.72	0.940
Medial-side surgery			
Nil (ref)	0		
Others	-0.74	-13.87, 12.39	0.912
Other medical condition			
Nil (ref)	0		
Seizure disorder	4.34	-2.99, 11.67	0.246
Others	1.49	-12.22, 15.21	0.831
Intraclass correlation (ICC): 0.47			
Tibiocalcaneal angle			
Age	-1.06	-2.05, -0.06	0.037
Follow-up surgery	0.99	0.37, 1.62	0.002
GMFCS			
2 (ref)	0		
3	-4.34	-14.36, 5.68	0.396
Medial-side surgery			
Nil (ref)	0		
Others	23.34	6.64, 40.04	0.006
Other medical condition			
Nil (ref)	0		
Seizure disorder	-0.93	-10.08, 8.21	0.841
Others	-26.70	-44.89, -8.50	0.004
Intraclass correlation (ICC): 0.00			
Talo-first metatarsal angle			
Age	-0.86	-2.10, 0.39	0.179
Follow-up surgery	0.15	-0.64, 0.94	0.713
GMFCS			
2 (ref)	0		
3	0.41	-12.18, 12.99	0.949
Medial-side surgery			
Nil (ref)	0		
Others	1.21	-19.32, 21.75	0.908
Other medical condition			
Nil (ref)	0		
Seizure disorder	-4.70	-16.21, 6.81	0.423
Others	-2.33	-23.55, 18.90	0.830
Intraclass correlation (ICC): 0.61			
Lateral talocalcaneal angle			
Age	-0.09	-0.86, 0.68	0.817
Follow-up surgery	0.21	-0.27, 0.70	0.388
GMFCS			
2 (ref)	0		
3	1.13	-6.66, 8.92	0.776
Medial-side surgery			
Nil (ref)	0		
Others	-2.04	-15.02, 10.95	0.758
Other medical condition			
Nil (ref)	0		
Seizure disorder	2.58	-4.53, 9.69	0.476
Others	0.93	-13.21, 15.07	0.897
Intraclass correlation (ICC): 0.00			
Naviculocuboid overlap			
Age	0.02	-0.09, 0.13	0.763
Follow-up surgery	0.01	-0.05, 0.08	0.688
GMFCS			
2 (ref)	0		
3	-0.76	-1.86, 0.35	0.181
Medial-side surgery			
Nil (ref)	0		
Others	0.09	-1.76, 1.94	0.925
Other medical condition			
Nil (ref)	0		
Seizure disorder	-0.99	-2.01, 0.01	0.053
Others	-0.17	-2.18, 1.84	0.867
Intraclass correlation (ICC): 0.00			
Metatarsal stacking angle			
Age	0.09	-0.47, 0.64	0.752
Follow-up surgery	0.35	0.001, 0.70	0.049
GMFCS			
2 (ref)	0		
3	0.23	-5.38, 5.84	0.936
Medial-side surgery			
Nil (ref)	0		
Others	-0.64	-9.99, 8.72	0.894
Other medical condition			
Nil (ref)	0		
Seizure disorder	-0.98	-6.11, 4.14	0.706
Others	-1.11	-11.30, 9.08	0.831
Intraclass correlation (ICC): 0.00			
Medial-lateral column ratio			
Age	-0.01	-0.01, 0.001	0.104
Follow-up surgery	-0.001	-0.01, 0.002	0.530
GMFCS			
2 (ref)	0		
3	-0.07	-0.13, -0.004	0.035
Medial-side surgery			
Nil (ref)	0		
Others	0.07	-0.03, 0.17	0.185
Other medical condition			
Nil (ref)	0		
Seizure disorder	-0.01	-0.07, 0.04	0.656
Others	-0.03	-0.14, 0.08	0.602
Intraclass correlation (ICC): 0.00			
Talonavicular coverage angle			
Age	1.22	-0.52, 2.97	0.170
Follow-up surgery	-0.38	-1.51, 0.74	0.501
GMFCS			
2 (ref)	0		
3	6.52	-13.33, 26.37	0.520
Medial-side surgery			
Nil (ref)	0		
Others	-8.56	-38.34, 21.22	0.573
Other medical condition			
Nil (ref)	0		
Seizure disorder	2.83	-15.87, 21.53	0.767
Others	-1.63	-32.79, 29.52	0.918
Intraclass correlation (ICC): 0.29			
First metatarsal talar angle			
Age	0.40	-1.61, 2.41	0.697
Follow-up surgery	-0.47	-1.76, 0.83	0.481
GMFCS			
2 (ref)	0		
3	-4.46	-27.16, 18.23	0.700
Medial-side surgery			
Nil (ref)	0		
Others	-1.87	-35.79, 32.04	0.914
Other medical condition			
Nil (ref)	0		
Seizure disorder	-13.18	-34.68, 8.32	0.230
Others	0.91	-33.69, 35.50	0.959
Intraclass correlation (ICC): 0.62			

RETRACTED

**Table 5:** Random intercept model: corrected feet GMFCS: Gross Motor Function Classification System

Variables	Odds ratio	95% CI	p-value
Calcaneal pitch			
Age	0.98	0.78, 1.23	0.841
Follow-up surgery	0.92	0.78, 1.07	0.277
GMFCS			
2 (ref)	1.00		
3	3.81	0.39, 37.39	0.252
Medial-side surgery			
Nil (ref)	1.00		
Others	0.10	0.003, 3.13	0.189
Intraclass correlation (ICC): 0.14			
Talo-first metatarsal angle			
Age	0.73	0.49, 1.07	0.109
Follow-up surgery	0.90	0.76, 1.07	0.255
GMFCS			
2 (ref)	1.00		
3	3.07	0.31, 30.79	0.340
Medial-side surgery			
Nil (ref)	1.00		
Others	1.56	0.12, 20.16	0.733
Intraclass correlation (ICC): 0.00			
Lateral talocalcaneal angle			
Age	1.27	0.94, 1.72	0.122
Follow-up surgery	0.97	0.82, 1.15	0.745
GMFCS			
2 (ref)	1.00		
3	2.56	0.28, 23.61	0.408
Medial-side surgery			
Nil (ref)	1.00		
Others	0.001	0.00, 21.11	0.049
Intraclass correlation (ICC): 0.00			
Naviculocuboid overlap			
Age	0.79	0.58, 1.08	0.135
Follow-up surgery	0.94	0.79, 1.12	0.495
GMFCS			
2 (ref)	1.00		
3	2.04	0.19, 21.84	0.557
Medial-side surgery			
Nil (ref)	1.00		
Others	6.79	0.05, 873.82	0.440
Intraclass correlation (ICC): 0.29			
Metatarsal stacking angle			
Age	0.78	0.60, 1.02	0.069
Follow-up surgery	1.06	0.90, 1.25	0.471
GMFCS			
2 (ref)	1.00		
3	0.66	0.08, 5.56	0.701
Medial-side surgery			
Nil (ref)	1.00		
Others	8.17	0.10, 646.57	0.346
Intraclass correlation (ICC): 0.00			
Talonavicular coverage angle			
Age	0.91	0.74, 1.12	0.373
Follow-up surgery	1.08	0.95, 1.23	0.243
GMFCS			
2 (ref)	1.00		
3	0.35	0.05, 2.33	0.278
Medial-side surgery			
Nil (ref)	1.00		
Others	19.26	0.41, 907.46	0.132
Intraclass correlation (ICC): 0.00			

## Discussion

The discussion section of the study provides a comprehensive analysis of the findings regarding the efficacy of CLO in correcting planovalgus deformity in pediatric patients with CP. It elucidates the associations between various factors and the outcomes of the surgical intervention, shedding light on potential implications for clinical practice and avenues for further research. One of the salient findings of the study is the statistically significant correction observed in the median calcaneal angle postoperatively, with approximately 35.5% of feet achieving normalization. This indicates that CLO holds promise as a viable surgical option for addressing planovalgus deformity in CP patients. The positive correlation between postoperative correction and factors, such as age, GMFCS level, and the presence of other medical conditions underscores the multifactorial nature of deformity correction in this population. Older children, particularly those with more severe functional impairment (as indicated by higher GMFCS levels) and comorbidities, may require more extensive correction, highlighting the importance of individualized treatment approaches.

RETRACTED

Conversely, the negative correlation between follow-up duration and the maintenance of correction suggests that long-term monitoring is crucial in assessing the durability of surgical outcomes. Over time, there may be a gradual loss of correction, necessitating periodic evaluations and, potentially, additional interventions to address recurrent deformities or complications. Furthermore, the study's identification of specific angles that showed significant differences between pre- and postoperative measurements provides valuable insights into the anatomical changes achieved through CLO, thereby enhancing our understanding of the surgical technique's biomechanical effects. The positive association between additional medial-side surgery and certain angles indicates that supplementary procedures may augment the corrective effects of CLO, particularly in cases where the deformity is more severe or multifaceted. However, it is essential to consider the potential risks and benefits of adjunctive interventions, weighing them against the overall treatment goals and patient-specific factors. Moreover, the negative correlations observed in children with seizure disorders and other medical conditions underscore the challenges inherent in managing complex cases with underlying medical complexities. These patients may present with more severe deformities or have limited tolerance for surgical interventions, necessitating a cautious approach and comprehensive preoperative assessment to optimize outcomes and minimize risks.

Comparing our study with the referenced research by Sung et al. [2] on surgical outcomes following CL procedures in pediatric cerebral palsy patients reveals nuanced similarities and differences. While both investigations demonstrate substantial improvements in foot and ankle alignment postoperatively, our study's slightly older patient cohort and shorter follow-up duration contrast with Sung et al.'s study, which involved a younger average age and longer follow-up period. Nevertheless, both studies observed significant enhancements in key angles, such as the AP talus-first metatarsal angle and naviculocuboid overlap, indicative of successful correction. Notably, Sung et al.'s study uniquely defined cutoff values for preoperative measurements, aiding in stratifying patients into corrected and undercorrected groups. These findings underscore the efficacy of CL procedures in addressing foot deformities in CP patients while emphasizing the importance of considering patient demographics and outcome measures in evaluating surgical success and guiding clinical decision-making. Further research integrating standardized outcome measures and larger patient cohorts is essential for refining surgical practices and optimizing long-term outcomes in this population [2].

RETRACTED

Comparing our study with Aboelenein et al.'s research [11] sheds light on similarities and differences in the outcomes of CL procedures for addressing planovalgus foot deformities in CP patients. Both investigations demonstrate significant improvements in radiographic measures following CL, with Aboelenein et al. reporting substantial enhancements in lateral talus-first metatarsal angle (Lat. T1MT), anteroposterior talus-first metatarsal angle (AP-T1MT), anteroposterior talocalcaneal angle (AP-TC), and lateral calcaneal pitch (Lat. CP). Similarly, our study observed major improvements in AP talus-first metatarsal angle, calcaneal pitch angle, talocalcaneal angle, lateral talus-first metatarsal angle, and naviculocuboid overlap post-CL. Both investigations also highlight the clinical efficacy of CL in relieving pain and correcting deformities in CP patients. However, differences emerge in reported clinical outcomes, with Aboelenein et al.'s study presenting detailed clinical improvement rates while our study focused on radiographic outcomes. Despite these disparities, both investigations affirm the effectiveness of CL in addressing pain and deformity in CP patients, providing valuable insights into the management of planovalgus foot deformities in this population [11].

Comparing our study with the research conducted by Cho et al. [18] on CL outcomes in patients with CP reveals several noteworthy similarities and distinctions. Both investigations aimed to assess radiographic outcomes following CL in CP patients, emphasizing the importance of clarifying indications and evaluating functional status in treatment decisions. However, notable differences exist in patient demographics and outcome measures. Our study included patients with a mean age of 11.0 ± 5.2 years and a minimum follow-up of 1.0 years (mean, 3.1 ± 2.2 years), whereas Cho et al.'s study involved patients with a slightly younger mean age of 10.5 ± 4.0 years and a longer mean follow-up of 5.1 ± 2.2 years. In addition, Cho et al.'s study specifically investigated the impact of the GMFCS level on outcomes, revealing that patients with GMFCS III/IV achieved less correction compared to those with GMFCS I/II. This finding contrasts with our study, which did not stratify outcomes based on the GMFCS level. Cho et al.'s study also identified a higher rate of undercorrection in GMFCS III/IV patients, suggesting the need for additional or alternative procedures to address deformity adequately. While both investigations underscore the efficacy of CL in correcting planovalgus foot deformities in CP patients, Cho et al.'s findings emphasize the importance of patient stratification based on the GMFCS level to optimize treatment outcomes and guide clinical decision-making effectively [18].

RETRACTED

It is crucial to recognize this study's limitations. First, the retrospective design brings inherent biases and limitations associated with collecting data retrospectively, including selection bias and incomplete or inconsistent data documentation. Moreover, the relatively small sample size might restrict the applicability of the findings and decrease the statistical power to identify significant associations. Furthermore, the study's reliance on radiographic measurements introduces the possibility of measurement errors and variability, which could impact the accuracy and reliability of the results. Lastly, the study's inclusion criteria and patient population, such as the predominance of male participants, may limit the extrapolation of findings to broader populations or diverse demographic groups. Future research endeavors should aim to address these limitations through prospective, multicenter studies with larger cohorts and comprehensive outcome assessments. Despite these limitations, this study makes a valuable contribution to our understanding and informs evidence-based practices in the surgical treatment of foot deformities associated with cerebral palsy.

## Conclusions

This study provides crucial insights into the efficacy of CLO for correcting planovalgus deformity in pediatric patients with CP. Our findings emphasize the multifaceted nature of deformity correction, highlighting the influential roles of age, GMFCS level, and comorbidities in shaping surgical outcomes. While CLO shows promise in achieving postoperative correction, our study underscores the importance of long-term follow-up to monitor the durability of correction and the potential for deformity recurrence. The identification of specific radiographic angles exhibiting significant changes postoperatively deepens our understanding of the biomechanical effects of CLO and provides valuable guidance for clinical decision-making. Moving forward, further research is warranted to elucidate optimal surgical approaches and refine patient selection criteria to maximize the benefits of CLO in this patient population.
